The article "Mapping of repeat-associated non-AUG (RAN) translation knowledge: A bibliometric analysis" was published in 2024. Journal: Heliyon.

# Mapping of repeat-associated non-AUG (RAN) translation knowledge: A bibliometric analysis

**DOI:** 10.1016/j.heliyon.2024.e29141

**Published:** 2024-04-02

**Authors:** Taiqi Zhao, Suying Duan, Jiaqi Li, Honglin Zheng, Chenyang Liu, Hang Zhang, Haiyang Luo, Yuming Xu

**Affiliations:** a Department of Neurology, The First Affiliated Hospital of Zhengzhou University, Zhengzhou University, Zhengzhou, Henan, China; b Henan Key Laboratory of Cerebrovascular Diseases, The First Affiliated Hospital of Zhengzhou University, Zhengzhou University, Zhengzhou, Henan, China; c The Academy of Medical Sciences of Zhengzhou University, Zhengzhou University, Zhengzhou, Henan, China; d Institute of Neuroscience, Zhengzhou University, Zhengzhou, Henan, China

**Keywords:** RAN translation, *C9orf72*, ALS, FTD, Small molecule, CiteSpace, VOSviewer, Bibliometric

## Abstract

Over 50 genetic human disorders are attributed to the irregular expansion of microsatellites. These expanded microsatellite sequences can experience bidirectional transcription, leading to new reading frames. Beyond the standard AUG initiation or adjacent start codons, they are translated into proteins characterized by disease-causing amino acid repeats through repeat-associated non-AUG translation. Despite its significance, there's a discernible gap in comprehensive and objective articles on RAN translation. This study endeavors to evaluate and delineate the contemporary landscape and progress of RAN translation research via a bibliometric analysis. We sourced literature on RAN translation from the Web of Science Core Collection. Utilizing two bibliometric analysis tools, CiteSpace and VOSviewer, we gauged individual impacts and interactions by examining annual publications, journals, co-cited journals, countries/regions, institutions, authors, and co-cited authors. Following this, we assessed the co-occurrence and bursts of keywords and co-cited references to pinpoint research hotspots and trending in RAN translation. Between 2011 and 2022, 1317 authors across 359 institutions from 34 countries/regions contributed to 250 publications on RAN translation, spread across 118 academic journals. This article presents a systematic, objective, and comprehensive analysis of the current literature on RAN translation. Our findings emphasize that mechanisms related to *C9orf72* ALS/FTD are pivotal topics in the realm of RAN translation, with cellular stress and the utilization of small molecule marking the trending research areas.

## 1 Introduction

Microsatellites, characterized by 3–6 bp repeat-sequence motifs, are alternatively termed simple sequences or short tandem repeats. These sequences are implicated in over 50 inherited human disorders. The expansion of microsatellite repeats instigates pathogenesis through three intertwined pathological mechanisms: protein loss-of-function, as well as RNA or protein gain-of-function. Over the past three decades, research into the pathogenesis of these aberrant microsatellite repeats has predominantly centered on their locational attributes. In non-coding domains, transcripts enriched with repeat expansions aggregate into RNA foci, sequestering specific RNA-binding proteins. Conversely, within AUG-initiated coding regions, they give rise to proteins in a unidirectional manner. Furthermore, the amplification of such repeats can influence *cis*-transcription, leading to the suppression of RNA and protein expression of the encompassing genes.

The unveiling of RAN translation upended traditional understandings of disease pathogenesis. Specifically, the expansion of microsatellites at the translational level, even without the presence of the AUG start codon, led to protein expression across multiple reading frames. In a seminal 2011 study, Zu et al. discerned that bidirectional transcripts of CAG and CUG repeat expansions can translate and facilitate proteins in all reading frames even in the absence of an AUG start codon. This atypical mode of translation was christened as repeat-associated non-AUG (RAN) translation [1]. It is now clear that RAN-translated proteins were found in multi-microsatellites associated with neurological diseases, such as *C9orf72* ALS/FTD, DM1, DM2, FXTAS, fragile X-associated primary ovarian insufficiency, fuchs endothelial corneal dystrophy, HD, SCA8, SCA31, and SCA36. RAN translation has blurred the mechanistic boundary between the coding and non-coding classifications. Whether or not it critically contributes to disease pathogenesis [2], proteins assumed to be amplified by microsatellite repeats and mutations previously thought to be non-coding and involved in RNA-mediated gain of function are now thought to be involved in diseases through RAN translation [[3], [4], [5]]. For example, RAN translation occurs at *C9orf72* in the coding strand-derived and antisense strand-derived repeat transcripts, generating five distinct dipeptide repeats from different reading frames [6,7]. In the cellular system, the RAN protein produced by *C9orf72* ALS/FTD generates key pathological features of *C9orf72* ALS/FTD by inhibiting adjacent cellular proteasome functions, leading to the misdistribution of tar DNA-binding protein 43 [8]. Since there are no effective treatments for microsatellite-expansion diseases, RAN translation has been considered a promising intervention point for various diseases. Moreover, numerous disorders linked to RAN-associated microsatellite expansions exhibit overlapping characteristics and pathogenic mechanisms. Progress in understanding pivotal aspects of this domain promises to illuminate research trajectories for related conditions.

A bibliometric analysis, both quantitative and qualitative, of extensive literature within a domain can illuminate insights on facets like countries, institutions, journals, references, authors, and keywords concurrently. This approach can unveil research hotspots and forecast impending research trajectories [[9], [10], [11]]. Compared to alternative analytical techniques, bibliometrics offers a more objective and dependable evaluation. Visual modeling through bibliometric scrutiny facilitates a methodical and exhaustive exploration of pivotal areas and innovations in a given field. Our investigation delves into the literature concerning RAN translation within the WOSCC database, with the intent to discern the current research landscape, pinpoint hotspots, and identify emerging research trends via bibliometric analysis.

In this article, we employ bibliometric techniques to classify, encapsulate, and visually represent pertinent RAN translation literature spanning from 2011 to 2022. We delve into the research advancements of RAN translation concerning neurogenetic degenerative ailments, including *C9orf72* ALS/FTD, HD, and FXTAS, illuminating prevailing research focal points and burgeoning perspectives within this domain. We underscore the significance of RAN translation in *C9orf72* ALS/FTD research and explore the nascent role of RAN proteins in gauging disease progression. Additionally, we touch upon the potential of small molecule interventions in RAN-associated microsatellite-expansion disorders, offering insights for future researchers.

## 2 Methods

### 2.1 Data collection

The search terms used to identify publications were (((TS = ("RAN translation")) OR TS = ("repeat-associated non-ATG translation")) OR TS = ("repeat-associated non-AUG translation")). The search was conducted in early 2023 for publications between 2011 and 2022. The bibliometric analysis data from the Web of Science Core Collection (WoSCC) search index included Science Citation Index Expanded (SCI-EXPANDED) and Social Science Citation Index (SSCI).

### 2.2 Inclusion criteria

Inclusion criteria were: (1) the literature related to RAN translation, including peer-reviewed original articles and reviews; (2) the languages are English.

### 2.3 Exclusion criteria

Exclusion criteria were: (1) publications involving plagiarism; (2) publications not officially published; (3) conference abstracts and proceedings and corrigendum documents; (4) unrelated publications.

### 2.4 Analysis methods and tools

In all, 250 publications were collected, including 182 original research articles and 68 review articles. The relevant information of all retrieved literature was exported and the bibliometric indicators were counted using Excel, including publication country/region, publication institution, the annual number of publications, citation frequency, average citation/publication frequency, journal name, the journal IF, SJR Indicator, author, and author's H-index. The retrieved studies were imported into CiteSpace (version 6.1.R6 advanced) and VOSviewer (version 1.6.18), to perform visualization analysis. CiteSpace was used to analyze details of the identified articles, including co-occurrence map of country/region and institutions, journals dual-map overlay, burst map, and timeline view of keywords. The CiteSpace parameters were as follows: Time Slicing (2011–2022), #Year Per Slice (1 year), Term Source (Title, Abstract, Author Keywords (DE), Keywords Plus (ID)), Node Types (Institution, Country or Keywords based on purpose), Pruning (Pathfinder, Pruning sliced networks and Pruning the merged network) and Visualization (Cluster view-static and Show merged network). VOSviewer was used to construct scientifically-based knowledge networks, including publication journals and co-cited journals, authors and co-cited authors, and keywords visualization.

## 3 Results

### 3.1 Outputs and bibliometric analysis by countries/regions and institutions

We have compiled the annual publications and citations of literature in this field over the past 12 years (Fig. 1). Over time, there was an overall increase in the number of publications. The first growth of publications was from 2012 to 2015 when the number of annual publications gradually increased from 1 to 21. The second growth was from 2018 to 2021 when there was a fierce increase in the annual number of publications. Citation rates have also increased over time, and have risen significantly since 2018.

**Fig. 1:** Annual number of publications and citations on RAN translation in the Web of Science from 2011 to 2022.

The retrieved 250 literature were from 34 countries/regions and 359 institutions (Table 1). The United States (*n* = 152, 60.8%) had the largest number of publications and citations, far exceeding the total number of publications from the four countries ranked after it, followed by England (*n* = 32, 12.8 %) and Germany (*n* = 27, 10.8%). The centrality of the United States, France, Spain, Japan, Germany, and Italy was above 0.10, suggesting “bridge” nodes in RAN translation studies. The United States (centrality = 0.93), France (centrality = 0.18), and Spain (centrality = 0.18) had high centrality values and are presented as purple circles in Fig. 2A. The University of Michigan (*n* = 29, centrality = 0.23), the University of Florida (*n* = 26, centrality = 0.14), and Mayo Clinic (*n* = 25, centrality = 0.35) had high production and centrality values (Fig. 2B). Country/region co-occurrence density (***ρ*** = 0.15) was above 0.1, which was an indication of active cooperation. However, the density of institutions co-occurrence (***ρ*** = 0.02) was under 0.1, indicating inactive cooperation among them.

**Table 1:** | Countries and regions’ publication number and citations.

Rank	Countries/Regions	Publications	Citations	Average Citation/Publication
1	the United States	152	9790	64.41
2	England	32	2122	66.31
3	Germany	27	2398	88.81
4	Japan	25	591	23.64
5	France	19	1860	97.89

**Fig. 2:** The co-occurrence map of countries/regions and institutions in RAN translation research. **(A)** Country/regions (n ≥ 1); **(B)** Institution (n ≥ 5). The node size reflects the co-occurrence frequencies, and the links indicate the co-occurrence relationships. The color of node and line represent different years; colors vary from gray to red as time goes from 2011 to 2022, and nodes with purple round mean high betweenness centrality (≥0.1). (For interpretation of the references to color in this figure legend, the reader is referred to the Web version of this article.)

### 3.2 Bibliometric analysis by journals and Co-cited journals

One Hundred and Eighteen journals published literature on RAN translation. Table 2 lists the top five journals that together published 62 literature, accounting for 24.8% of all literature published, with *Human Molecular Genetics* publishing the largest number of literature (*n* = 15), while *Neuron* generated the highest citation/publication ratio (*n* = 14, *r* = 213.86).

**Table 2:** | Number of publications from the top five journals.

Rank	Journal	Publications	Citations	Average Citation/Publication	IF(2022)	JCR(2022)
1	Human Molecular Genetics	15	753	50.2	3.5	Q1
2	Neuron	14	2994	213.86	16.2	Q1
3	Acta Neuropathologica Communications	13	257	19.77	7.1	Q1
4	Acta Neuropathologica	12	1964	163.67	12.7	Q1
5	Journal of Biological Chemistry	8	494	61.75	4.8	Q1

Co-cited journals are different journals simultaneously served as sources of literature in the references of articles. Among the 1222 co-cited sources, 36 had more than 100 citations. The top 10 co-cited journals that accounted for 86.9% of all cited references are listed in Table 3. Among them, *Neuron* (*n* = 1520), *Human Molecular Genetics* (*n* = 1164), and *Acta Neuropathologica* (*n* = 1047) were the most cited. We selected 36 co-cited journals according to the minimum number of relevant publications (*n* = 100) and plotted a co-cited journal network map (Fig. 3).

**Table 3:** | Top 10 co-cited journals.

Rank	Cited journal	Co-citations	JCR(2022)	IF(2022)
1	Neuron	1520	Q1	16.2
2	Human Molecular Genetics	1164	Q1	3.5
3	Acta Neuropathologica	1047	Q1	12.7
4	PNAS	926	Q1	11.1
5	Science	871	Q1	56.9
6	Nature	677	Q1	64.8
7	Cell	616	Q1	64.5
8	Nucleic Acids Research	607	Q1	14.9
9	Journal of Biological Chemistry	566	Q1	4.8
10	Molecular Cell	349	Q1	16

**Fig. 3:** The network map showing co-cited journals (n ≥ 100) that have published research on RAN translation.

The journal dual-map overlay shows the topic distribution among academic journals [12] (Fig. 4). The literature was categorized into two groups using a dual-map overlay: (1) cited journals and (2) citing journals. The latter refers to journals that cited their references from the former. Through the use of journal co-citation analysis, dual-map overlay can effectively illustrate the relationship between the distributions of cited journals and citing journals in the literature. The figure shows that there was only one primary citation's path, from MOLECULAR/BIOLOGY/IMMUNOLOGY journals to MOLECULAR/BIOLOGY/GENETICS journals.

**Fig. 4:** The dual-map overlay of journals on RAN translation. The citing journals are on the left, and the cited journals are on the right. The colored path represents the citation relationship.

### 3.3 Bibliometric analysis of authors and Co-cited authors

A total of 1317 authors were involved in RAN translation publications, of which 36 published at least five literature. Todd, PK. (*n* = 26, H-index = 29) was a co-author of the largest number of RAN translation-related literature, followed by Petrucelli, L (*n* = 21, H-index = 80) and Ranum, Laura P. W. (*n* = 21, H-index = 54; Table 4). Petrucelli, L from the Mayo Clinic in Jacksonville, Florida, was undoubtedly the most influential and contributing author in terms of the number of publications and citations. ‘Unconventional translation of *C9orf7*2 GGGGCC expansion generates insoluble polypeptides specific to c9FTD/ALS’ was this author's most cited article in this field. It describes the generation of insoluble proteins specific to *C9orf72*-mediated FTD/ALS by RAN translation of the GGGGCC repeats in *C9orf72* [13]. Todd, PK. from the University of Michigan, Ann Arbor, Michigan, and Ranum, Laura P. W. from the University of Florida, Gainesville, Florida, also had a considerable influence in the field.

**Table 4:** | Top 5 co-authors related to the RAN translation field.

Rank	Co-author	Publication	Citations	H-index
1	Todd, PK.	26	1059	29
2	Petrucelli, L	21	3585	80
3	Ranum, Laura P. W.	21	2315	54
4	Gendron, TF.	16	2249	50
5	Krans, A	14	660	11

Co-cited authors are different first authors in the references of articles. Among the 7351 co-cited authors, 39 had over 50 co-citations. Fig. 5 presents the co-cited authors as a density plot, clearly showing the high-frequency co-cited authors. Table 5 and Fig. 5 show that Zu, T (*n* = 334, H-index = 17), Mori, K (*n* = 258, H-index = 17), and Sellier, C (*n* = 176, H-index = 19) had the highest number of co-citations.

**Fig. 5:** The density visualization map of co-cited authors (n ≥ 50) in the RAN translation field. The size of the word and the opacity of yellow are positively related to the co-cited frequency. (For interpretation of the references to color in this figure legend, the reader is referred to the Web version of this article.)

**Table 5:** | Top 5 co-cited authors related to the RAN translation field.

Rank	Co-cited Author	Co-citations	H-index
1	Zu, T	334	17
2	Mori, K	258	17
3	Sellier, C	176	19
4	Todd, PK.	155	29
5	Zhang, YJ	147	27

### 3.4 Bibliometric analysis of Co-cited references and reference bursts

Among the 9597 citations, 27 articles were cited at least 50 times (Fig. 6A). Co-cited references are two or more articles simultaneously cited by other articles. Table 6 summarizes the top five co-cited references, with the least cited 120 times. The most cited article was by Zu T et al. demonstrating that RAN translation not only in cell culture models but also in human disease for the first time [1]. This report demonstrates that RAN proteins accumulate not only in cells with CAG expansion constructs but also in patient tissues from both SCA8 and DM1. This significant finding has led to the identification of RAN translation in *C9orf72* ALS/FTD and other related disorders. Furthermore, four of the five most cited articles focused on *C9orf72*, while the fifth explained the RAN translation mechanism. It is evident that *C9orf72* has a significant impact in the field of RAN translation.

**Fig. 6:** **(A)** The network map of co-cited references related to RAN translation; **(B)** Top 25 references with the strongest citation bursts.

**Table 6:** | Top five co-cited references related to RAN translation.

Rank	Title	First Author	Journals	Co-cited Counts	Year
1	Non-ATG-initiated translation directed by microsatellite expansions	Zu, T	PNAS	152	2011
2	Unconventional translation of C9ORF72 GGGGCC expansion generates insoluble polypeptides specific to c9FTD/ALS	Ash, Peter E. A.	Neuron	139	2013
3	Expanded GGGGCC hexanucleotide repeat in noncoding region of C9ORF72 causes chromosome 9p-linked FTD and ALS	DeJesus-Hernandez, M	Neuron	139	2011
4	The C9orf72 GGGGCC repeat is translated into aggregating dipeptide-repeat proteins in FTLD/ALS	Mori, K	Science	136	2013
5	A hexanucleotide repeat expansion in C9ORF72 is the cause of chromosome 9p21-linked ALS-FTD	Renton, AE.	Neuron	133	2011

Citation bursts are defined as publications cited significantly more often for a while, in which the most frequently cited are considered to be the basis for the direction of the frontier in a given field. The 25 publications with the strongest citation burst are listed in Fig. 6B. The highest and second highest citation burst references were generated by DeJesus-Hernandez et al. and Renton et al. These authors identified a non-coding expanded GGGGCC hexanucleotide repeat in *C9orf72* as the cause of chromosome 9p-linked ALS/FTD and showed that this genetic defect is the most common cause of ALS and FTD [14,15]. Besides, they proposed the concept of *C9orf72* ALS/FTD. According to the analysis of citation burst, we can find that research on the molecular mechanisms involved in *C9orf7*2 RAN translation and interventions are hot topics. Among the publications whose bursts lasted until 2022, more than half were about the *C9orf7*2 RAN translation. These cited studies are seminal publications in the field, and they provide the basis for studies to follow.

### 3.5 Bibliometric keyword analysis

We extracted 1131 keywords and used VOSviewer to analyze those appearing >10 times. Table 7 lists the top ten keyword co-occurrences, and Fig. 7A shows the high-frequency keywords (>10 times) as an overlay map. Small molecule, CGG repeats, in-vitro, and mouse model were emerging fields, colored in yellow in the figure. Three keyword clusters were noted in the cluster visualization map (Fig. 7B). Duplicate keywords were removed using Thesaurus (Supplementary_Table_S1), such as als or amyotrophic lateral sclerosis were replaced by amyotrophic-lateral-sclerosis. The keywords in each cluster were strongly interrelated. Keywords in the green cluster included *C9orf72*, FTD, ALS, TDP-43, GGGGCC repeat, RNA foci, and hexanucleotide repeat expansion. The blue cluster included keywords such as small molecules, drosophila, in-vitro, protein, expansion, and expression. The red cluster included keywords such as translation, in-vivo, fmr1 messenger-RNA, myotonic-dystrophy, mouse model, CGG repeat, intranuclear inclusions, and FXTAS. These clusters indicate that studies centered on *C9orf72*, ALS, hexanucleotide repeat expansion, translation, RNA foci, small molecule, and in-vitro are the current focus in RAN translation research.

**Table 7:** | Top 10 co-occurrence times of keywords.

Rank	Counts	Keywords	Link Strength
1	131	translation	683
2	103	amyotrophic lateral sclerosis	649
3	89	C9orf72	577
4	86	hexanucleotide repeat expansion	517
5	58	RNA foci	405
6	57	neurodegeneration	333
7	54	protein	303
8	50	antisense transcripts	352
9	48	expansion	286
10	46	frontotemporal lobar degeneration	306

**Fig. 7:** **(A)** The overlay map of keywords based on VOSviewer. The color represents the average year of publication; **(B)** The cluster visualization map of keywords based on VOSviewer. (For interpretation of the references to color in this figure legend, the reader is referred to the Web version of this article.)

The timeline view (Fig. 8) presents high-frequency keywords in each cluster over time. Seven of the eleven clusters (except #3, #4, #9, and #10) are still in progress. Among them, cluster #0 (motor neuron disease) was the largest, followed by #1 (neuron), #2 (small molecule), #5 (parent-of-origin effect), #6 (polyglutamine diseases), #7 (*c9orf72* repeat expansion mutation) and #8(liquid-liquid phase separation).

**Fig. 8:** The timeline view of keywords. Each horizontal line represents a cluster, and the threshold for the number of articles in each cluster is 10. The smaller the number, the larger the cluster, and #0 is the largest. The time is at the top, and keywords are located at their first co-occurrence time in the cluster. Cluster labels were extracted from the title and abstract information by MI analysis and nodes with purple round mean high betweenness centrality (≥0.1). Harmonic Mean (Q, S) = 0.87 > 0.80, indicating that clustering was considered credible. MI, mutual information. (For interpretation of the references to color in this figure legend, the reader is referred to the Web version of this article.)

Keyword bursts are keywords that are frequently cited over time [16]. We used CiteSpace to detect the top 10 burst keywords with the largest number of citations during 2011–2022 (Fig. 9). The figure ranks the keywords according to the beginning year of burst. Keywords with high burst values (>3.00) imply high research attention and influence in the corresponding period. As shown in the figure, frontotemporal lobar degeneration had the strongest burst (6.02). It can be found that frontotemporal lobar degeneration, *C9orf72* hexanucleotide repeat, and antisense transcript emerged as early research directions from 2013 to 2015, consistent with the trend of citation burst. The keywords with high burst values between 2016 and 2018 are tremor ataxia syndrome and nucleocytoplasmic transport. There are keywords such as in vitro, small molecule, and mouse model which continued to 2022.

**Fig. 9:** Top ten keywords with the strongest citation bursts from 2011 to 2022. The red bars represent the years in which the keywords were used most frequently and the green bars represent the years in which the keywords were used least frequently. (For interpretation of the references to color in this figure legend, the reader is referred to the Web version of this article.)

## 4 Discussion

### 4.1 General information

Based on the 2011–2022 data retrieved from the WoSCC database, 250 RAN translation publications were published in 118 academic journals by 1317 authors in 359 institutions from 34 countries/regions. A growing body of literature indicates that RAN translation is attracting increasing attention and interest. More importantly, the analysis of research hotspot diseases may provide new research ideas for other diseases that also serve as RAN-associated microsatellite-expansion disorders. The RAN translation research started in 2011 when Zu et al. proposed the term [1]. Since then, RAN translation research has grown rapidly.

An analysis by country/region revealed that the United States and its affiliated institutions were the predominant contributors to publications on RAN translation (Table 1). Researchers from the United States not only produced the most publications but also garnered the highest number of citations. Intriguingly, France led in terms of average citations per publication. Nodes with a high centrality (≥0.10) serve as "bridges" in the global cooperation network, as delineated in Refs. [17,18]. According to Table 1 and Fig. 2A, nations such as the United States, France, Japan, and Germany exhibited both high publication counts and betweenness centrality, underscoring their pivotal roles in fostering global collaboration in RAN translation studies. However, the sparse inter-institutional cooperation observed in co-occurrence plots suggests a pressing need to bolster collaborative efforts.

Upon analyzing journals and authors, it became evident that *Neuron* stands as a cornerstone in the field. Not only is it the most frequently cited journal, but it also holds the second rank in terms of publications. Remarkably, three out of the top five most-cited articles found their home in this journal [[13], [14], [15]]. Both *Human Molecular Genetics* and *Acta Neuropathologica* are among the top five in terms of impact and citations, underscoring their pivotal roles in propagating RAN translation research. These esteemed journals predominantly delve into areas of molecular biology, immunology, and genetics. Notably, Todd, PK. has graced the field with the most substantial volume of literature and stands as one of the top five most-cited authors.

Reference analysis (Fig. 6B) indicated that DeJesus-Hernandez, M; Renton, AE.; Zu, T; Ash, Peter E. A.; Mori, K; Green, KM.; Cheng, W were the most cited authors, showing outbreak intensity that deserves to be studied in depth by novice researchers in this field [1,14,15,19]. Green, KM.; Cheng, W; Zhang, YJ; Shi, Y; Sonobe, Y; Tabet, R; Westergard, T published burst literature that continues to be cited until 2022, helping to find the hotspots in this field [[20], [21], [22], [23], [24], [25]].

### 4.2 The hotspots and trending

In an age saturated with information, it's imperative for researchers to stay attuned to the evolving research landscapes in their domain. Within bibliometrics, the interplay of keyword co-occurrence and bursts offers insights into the foundational content and trending research areas of a scholarly subject [16,26]. The overlay and timeline perspectives shed light on the emergence of research hotspots [27,28], while citation bursts delineate the nascent topics gaining traction in the field [16]. In this study, we tried to objectively evaluate the hotspots and trending of RAN translation research through the analysis of citation bursts (Fig. 6B), keyword co-occurrence (Table 7), visualization map (Fig. 7), timeline view (Fig. 8), and keyword bursts (Fig. 9).

By summarizing the results of the related analyses, it can be concluded that the main focus of RAN translation research is on the mechanisms related to *C9orf72* ALS/FTD. The research trend gradually shifts from observing phenomena to investigating underlying mechanisms, with the ultimate goal of clinical application. The advancement in *C9orf72* ALS/FTD research serves as a valuable reference for exploring RAN translation in other neurodegenerative diseases. We summarized the hotspots and trending research areas as follows.

#### 4.2.1 Mechanisms of RAN translation in neurodegenerative diseases

According to keyword analysis and citation bursts, research into RAN translation-related neurodegenerative diseases is an important investigation focus. It included specific diseases (i.e., ALS, FTD, HD, FXTAS) and related pathological mechanisms (i.e., RAN translation, *C9orf72* hexanucleotide repeat, antisense transcript, nucleocytoplasmic transport, CAG repeats, RNA foci, antisense RNA, CGG repeats, and liquid-liquid phase separation). These results illustrated that research hotspots were mainly focused on the mechanisms of RAN translation in various neurodegenerative diseases. Our results identified *C9orf72* ALS/FTD-related mechanisms as a hotspot in the field of RAN translation, whereas cellular stress is a current research frontier.

Through a meticulous analysis of citation bursts, it becomes evident that mechanisms related to *C9orf7*2 RAN translation are undeniably at the epicenter of RAN translation research. This observation aligns seamlessly with the outcomes of our keyword analysis. The intricacies of *C9orf72* ALS/FTD RAN translation and its affiliated pathological mechanisms have been extensively probed. A pivotal moment in this realm was in 2011 when multiple research cohorts, almost in synchrony, pinpointed a GGGGCC hexanucleotide repeat expansion in the non-coding precinct of *C9orf72* as the catalyst for chromosome 9p-linked ALS/FTD [14,15,29]. Studies at that time only found that the upstream hexanucleotide repeat expansion affected the downstream normal *C9orf72* protein expression by inhibiting transcription (protein loss of function) and by generating toxic RNA foci (RNA gain of function).

It wasn't until 2013 that the significance of bidirectional transcription and RAN translation emerged as pivotal pathological hallmarks of *C9orf72* ALS/FTD. Employing an antibody specifically tailored against the conjectured GGGGCC repeat RAN translation peptide (dubbed anti-C9RANT), Peter et al. discerned the presence of high molecular weight insoluble constituents in brain samples from familial ALS/FTD patients [13]. Moreover, intraneuronal inclusions were ubiquitously observed throughout the central nervous system. Notably, inclusion bodies extracted from patient tissues were laden with poly(Gly-Ala), poly(Gly-Pro), and poly(Gly-Arg) dipeptide repeat proteins [19]. The GGGGCC hexanucleotide repeat expansion in familial ALS/FTD was found to instigate the synthesis of both sense and antisense RNAs, leading to the accumulation of five distinct RAN proteins [6,7]. These proteins are the byproducts of RAN translation occurring across three reading frames. In a subsequent exploration, leveraging a neuronal model derived from patient-specific induced pluripotent stem cell differentiation, it was discerned that RNA foci disrupt the innate physiological harmony of cells. This disruption is attributed to the sequestration of RNA-binding proteins like hnRNPA1, Pur-α, and ADARB2 within neurons [30,31]. Remarkably, antisense oligonucleotide treatments aimed at the *C9orf72* transcription product have shown promise in inhibiting RNA foci formation in neurons, thereby mitigating the pathological aberrations induced by RNA protein expression.

Subsequent investigations have delved deeply into the pathological mechanisms by which RAN proteins instigate *C9orf72* ALS/FTD. In 2014, through the development of a drosophila model that expressed unadulterated repetitive sequences, Mizielinska et al. and Kwon et al. found that both arginine-rich proteins and RNA-containing repeat expansions contribute to *C9orf72*-mediated neurodegeneration, while dipeptide repeat proteins (DPRs) are the main toxic species [32,33]. In neuronal models, it was discerned that arginine-rich dipeptide repeat proteins, especially poly(Pro-Arg), exhibited neurotoxic properties [34]. Poly(Pro-Arg) aggregates in the nucleolus, leading to a decrease in the RNA processing body and the formation of stress granules, suggesting that global cellular translation dysregulation is a major pathway of toxicity produced by RAN proteins. Advancing this understanding, in 2015, Freibaum et al. crafted drosophila models expressing varying lengths of GGGGCC repeat expansions, mirroring those found in patient neural tissues. Their observations revealed a dose-responsive, repeat length-specific neurodegeneration, accompanied by RAN translation of dipeptide repeat proteins in these genetically modified organisms [35]. Intriguingly, RAN proteins interfere with the nuclear pore complex, resulting in a dysfunctional mechanism that coordinates nuclear RNA export and nuclear protein import. Application of the small molecule RanGAP (drosophila ortholog of human RanGAP1), the key regulator of nucleocytoplasmic transport in the nucleus, inhibited neurodegeneration in a drosophila model with GGGGCC repeat sequence by enhancing nuclear inputs and inhibiting nuclear outputs [36].

Analyzing citation bursts from recent years can provide valuable insights into the forefront of research. Green and colleagues pinpointed that changes in start codon fidelity, dependent on eIF2α phosphorylation, amplified both *C9orf7*2 RAN and CGG RAN. Interestingly, the formation of stress granules reliant on phosphorylated eIF2α and the overarching inhibition of translation were consistently triggered by both CGG and GGGGCC repeats [20]. RAN translation sees an upsurge when the phosphorylation of the eukaryotic initiation factor-2 (eIF2α) is stimulated by diverse stressors. Moreover, compounds that curtail the phosphorylated eIF2α pathway have demonstrated an ability to inhibit RAN translation [21]. These revelations bolster the theory of a feed-forward loop model. Within this framework, repeat expansion instigates cellular stress conditions conducive to RAN translation of deleterious proteins. This, in turn, produces an influx of dipeptide repeat proteins by assimilating the stress response, further accelerating the onset of neurodegeneration. Notably, antibodies aimed at RAN proteins have shown efficacy in diminishing protein aggregates, subsequently improving behavior and mitigating neurodegeneration in *C9orf7*2 BAC mice [37].

From our analysis of the keyword timeline view and visualization map, the CAG trinucleotide repeat expansion in HD emerged as a significant point of interest. HD is characterized as a neurodegenerative ailment, stemming from the CAG trinucleotide repeat expansion within the huntingtin gene. In addition to polyGln expansion proteins, four novel homopolymeric expansion proteins (polyAla, polySer, polyLeu, and polyCys) were identified in patient-derived tissues. Elevated levels of HD-RAN proteins, coupled with the death of neuronal and glial cells, have been observed in cellular models [38,39]. Such findings corroborate the presence of bidirectional transcription and RAN translation in HD. According to a study conducted by Su Yang et al., it was observed that RAN translation is not detected in the knock-in mouse models when expanded CAG repeats are expressed at the endogenous level [2]. The researchers suggested that RAN-translated products do not significantly contribute to the pathogenesis of CAG repeat diseases. Intriguingly, while the onset of HD is contingent upon the size of continuous CAG repeats rather than polyglutamine, the inception and progression of the disease can be anticipated and tracked. This can be achieved by monitoring RAN proteins, alongside cerebrospinal fluid and serum biomarkers such as the neurofilament light chain and the mutant protein [40,41].

Further insights from the overlay map analysis spotlight the significance of the terms “FXTAS” and “CGG repeats”. The CGG repeat expansions located in the 5′UTR of *FMR1* lead to the synthesis of polyglycine-rich proteins, termed FMRpolyG, through RAN translation. This process is responsible for a neurodegenerative disorder known as FXTAS. It has been observed that FMRpolyG adversely impacts neuronal cells, disrupting laminin anchoring, inducing mitochondrial anomalies, and precipitating cellular degradation [42,43]. Research by Asamitsu et al. revealed that CGG-G4 RNA has a direct affinity to the polyglycine segment of FMRpolyG, facilitating the emergence of aggregates stemming from liquid-liquid phase separation. Additionally, FMRpolyG is channeled into exosomes, enabling intercellular transfer and leading to neuronal disturbances. A notable intervention, the oral intake of PpIX-convertible 5-ALA, has demonstrated efficacy in alleviating synaptic malfunctions and behavioral challenges in CGG-KI mice. This is achieved by suppressing the expression and clustering of the FMRpolyG RAN protein [44]. An intriguing +1 translational frameshift occurring within the initial set of translated CGG repeats causes a reading frame transition from arginine (R) to glycine (G). This results in the formation of truncated chimeric R/G peptide aggregates, which exhibit toxic properties in rodent neuron cultures [45]. A landmark discovery in FXTAS research highlighted that the neurotoxic protein FMRPolyG can be quantified in samples sourced from humans. This mechanism, intertwined with RAN translation, offers a pioneering instrument for preemptive disease detection [46].

The bibliometric analysis tool offers a gateway to articles that have garnered significant citations across various timeframes. Delving into these articles equips researchers with a comprehensive knowledge landscape. Within the realm of RAN translation, our findings underscore that research related to *C9orf72* ALS/FTD RAN translation stands out as a focal point. By examining highly cited articles spanning different eras, it becomes evident that bidirectional transcription and the formation of RAN proteins are foundational pathological characteristics. These elements engender cytotoxicity through mechanisms such as the segregation of RNA-binding proteins, disruption of nucleoplasmic translocation, and the onset of cellular stress. Concentrating on *C9orf72* ALS/FTD research promises to unveil fresh insights into the mechanisms underlying other RAN-associated microsatellite-expansion disorders. Moreover, it holds the potential to identify innovative avenues for therapeutic development.

#### 4.2.2 New intervention targets: application of small molecule

Keyword bursts spotlight “in-vitro”, “small molecule”, and “mouse model” as emerging research trends. Concurrently, the term “small molecule” features prominently in both the overlay map and timeline view, marking its significance in recent publications and as a distinct research cluster. Given these observations, it's evident that targeting RAN translation via small molecule is poised to be a pivotal research direction. Regrettably, drug development does not always proceed without obstacles. An investigational antisense oligonucleotide BIIB078, which was intended to treat *C9orf72* ALS, did not demonstrate clinical efficacy. Furthermore, clinical trials have shown that certain antisense oligonucleotide drug candidates targeting HTT mRNA have also proven unsuccessful [47]. The therapeutic form of antisense oligonucleotides is still in its infancy. Thus, there's a pressing need for innovative therapeutic strategies for RAN-associated microsatellite-expansion disorders. Our findings underscore that the primary targets for small molecules in these disorders encompass both the toxic function of expanded RNA and the toxic function of repeat expansion proteins.

In *C9orf72* ALS/FTD, the expanded GGGGCC RNA adopts two folding states in equilibrium: the hairpin structure and the G-quadruplex. Bioactive small molecules targeting the expanded RNA have demonstrated significant inhibition of RAN translation and the formation of RNA foci in cultured cells expressing GGGGCC repeats and in patient-derived fibroblasts [48,49]. A small molecule, CB253, has the capability to selectively bind to hexanucleotide repeats that amplify GGGGCC in a specific conformation found in *C9orf72* ALS/FTD [50]. In a recent study of *C9orf72* ALS/FTD, it was discovered that the nucleoside analog decitabine eliminated RNA foci within the GGGGCC repeat without affecting the entire gene expression. This approach also led to a reduction in dipeptide repeat sequences and an attenuation of pathology in transgenic mice [51]. Furthermore, HSP90 inhibitor geldanamycin and aldosterone antagonist spironolactone have been shown to promote protein degradation, reduce dipeptide repeat protein levels, and reverse the pathological phenotype in the *C9orf72* ALS/FTD Drosophila model [52].

Intervention against the toxicity of dipeptide repeat proteins is also at the forefront of research in the field of RAN translation. As previously explained, RAN translation initiates a feed-forward loop pathway wherein the dipeptide repeat protein generated by RAN translation triggers the up-regulation of the integrated stress response. This, in turn, leads to increased RAN translation. Consequently, inhibitors of the integrated stress response, such as ISRIB, and other small molecules that target the endoplasmic reticulum stress response, hold promise as potential therapeutic strategies for addressing *C9orf72* ALS/FTD. These approaches have the potential to disrupt this detrimental feed-forward loop [21,53].

Inspired by studies related to *C9orf72* ALS/FTD, the application of small molecule in FXTAS has also garnered significant attention. Natural bioactive small molecules like curcumin and piperine, by selectively recognizing CGG repeat RNA, have shown the ability to ameliorate FXTAS-associated selective splicing defects and reduce the production and accumulation of FMRpolyG protein inclusion bodies [54,55]. In addition, 5-aminolevulinic acid has been found to improve aberrant synaptic plasticity and behavior in the FXTAS mouse model. This is achieved by inhibiting RAN translation and liquid-liquid phase separation [44]. Furthermore, small molecules like 1a and lead molecules B1, B4, and B11 have demonstrated the capacity to protect CGG repeat-amplified RNA and reduce the levels of FMRPolyG-positive aggregates, without progression toward FXTAS pathology [56,57]. Moreover, the serine/arginine protein kinase inhibitor, SRSF protein kinase 1, has been effective in inhibiting RAN translation of both GGGGCC and CGG repeats. It has also shown the ability to suppress toxicity in a *C9orf72* ALS/FTD Drosophila model and in CGG repeat-bearing rodent neurons. Consequently, these inhibitors hold promise as a novel treatment for both *C9orf72* ALS/FTD and FXTAS, both of which are caused by RAN translation of aberrantly amplified microsatellites [58]. The application of small molecule to target RAN translation has demonstrated significant therapeutic potential for neurodegenerative diseases, which has attracted the interest of researchers and has become a promising area of research.

### 4.3 Strengths and limitations

This was the first bibliometric study to systematically analyze the RAN translation literature and its development trends intuitively, objectively, and accurately, providing comprehensive guidance for clinicians and related scholars. The bibliometric analysis provides valuable and objective insights into the evolving research foci and trends. This study will inform the public of the importance of RAN translation-related diseases, provide scholars with a thorough picture of RAN translation research, and serve as a comprehensive and objective guide for future developments in the field.

Inevitably, this study had some limitations. First, our study exclusively retrieved literature published in English from the WoSCC database; data from other important databases were excluded, and some linguistic bias may have been introduced. Second, bibliometric methods are based on natural language processing, which might be biased, as reported by others [59].

## 5 Conclusion

Currently, there are exciting developments in the field of RAN translation, and our understanding of RAN translation has improved dramatically over the past 12 years. The current research focus on *C9orf72* ALS/FTD is critical to advancing our understanding of RAN-associated microsatellite-expansion disorders from observing research phenomena to exploring mechanisms, ultimately leading to clinical applications. Our results suggest that impaired nucleocytoplasmic transport and cellular stress are pathogenic mechanisms of interest, while repeat toxic RNA and proteins are valuable intervention targets. The bibliometric and visualized analysis will help to obtain the current state of the scientific research in a given field, with the advantage of qualitative and quantitative access to the hot research contents and cutting-edge directions. Many RAN-associated microsatellite-expansion disorders share common pathological mechanisms, such as the hairpin structure and the G-quadruplex of repeat RNA and RAN protein generation. It is our belief that the current state of research in hotspots will inspire researchers to explore similar disorders.

## Fundings

The author(s) disclosed receipt of the following financial support for the research, authorship, and/or publication of this article: The author's work was supported by the 10.13039/501100001809National Natural Science Foundation of China (Grant U1904207 to Dr. Yuming Xu) and the Non-profit Central Research Institute Fund of 10.13039/501100005150Chinese Academy of Medical Sciences (Grant 2020-PT310-01 to Dr. Yuming Xu).

## Ethics statement

Informed consent was not required for this study because all data used were obtained from the Web of Science database.

## Data availability statement

Data included in article/supp. material/referenced in article.

## CRediT authorship contribution statement

**Taiqi Zhao:** Visualization, Writing – original draft. **Suying Duan:** Writing – review & editing. **Jiaqi Li:** Visualization, Writing – review & editing. **Honglin Zheng:** Writing – review & editing. **Chenyang Liu:** Writing – review & editing. **Hang Zhang:** Visualization. **Haiyang Luo:** Conceptualization, Writing – review & editing. **Yuming Xu:** Conceptualization, Writing – review & editing.

## Declaration of competing interest

We declare that we have no financial and personal relationships with other people or organizations that can inappropriately influence our work, there is no professional or other personal interest of any nature or kind in any product, service and/or company that could be construed as influencing the position presented in, or the review of, the manuscript entitled.
